This article has been retracted.

# Clinical Characteristics and Death Risk Factors of Severe Sepsis in Children

**DOI:** 10.1155/2022/4200605

**Published:** 2022-01-24

**Authors:** Ying Zhang, Buqing Cao, Weihong Cao, Hongjun Miao, Lihui Wu

**Affiliations:** ^1^Department of Neonatology, Xiangyang No.1 People's Hospital, Hubei University of Medicine, Xiangyang, Hubei 441000, China; ^2^Department of Laboratory Medicine, Ruikang Hospital Affiliated to Guangxi University of Chinese Medicine, Nanning, Guangxi 530001, China; ^3^Department of Pediatrics, Affiliated Renhe Hospital of China Three Gorges University, Yichang, Hubei 443000, China; ^4^Emergency Department, Children's Hospital of Nanjing Medical University, Nanjing, Jiangsu 210008, China

## Abstract

Sepsis is a systemic inflammatory response syndrome caused by viral infection. The circulatory dysfunction caused by sepsis is also called septic shock or septic shock. The main characteristics are rapid onset, rapid changes, and involvement. Multiple organs in the body make diagnosis difficult, which seriously threatens the survival of patients. As many as one million people worldwide die every year because of SIRS, it is also the leading cause of death among children in hospital ICUs. This article is aimed at studying the clinical characteristics of severe sepsis in children and the risk factors for death. Based on the analysis of the pathogenesis of sepsis and the treatment of septic shock, 65 cases of children with PICU sepsis admitted to a hospital were selected. Data, to study its clinical characteristics and risk factors for death. The results of the study showed that despite the interaction among the removal factors of the three indexes of serum lactic acid value, PCIS level, and the number of organs involved in MODS, they are still related to the mortality of children with severe sepsis.

## 1. Introduction

Sepsis is a syndrome of body inflammation caused by various suspected or proven infectious pathogens. Severe sepsis refers to tissue infiltration and/or multiple organ dysfunction caused by sepsis [1, 2]. The incidence of PICU sepsis and severe sepsis in China is gradually increasing, and the mortality rate is also on the rise [3, 4]. Sepsis, severe sepsis, and septic shock can be divided according to the severity of sepsis. Severe sepsis refers to sepsis accompanied by organ dysfunction, poor tissue perfusion, or hypotension. Septic shock is a special type of severe sepsis, which is still accompanied by uncorrectable continuous hypotension after sufficient fluid resuscitation.

Sepsis is caused by the body's disordered host response to viral infections, which threatens survival with multiple organ dysfunction syndrome. The occurrence and onset of sepsis are a highly complex pathological and biological process, including many mechanisms, such as hemodynamic disorders and anti-inflammatory and proinflammatory dysfunction. Current studies have confirmed that the main cause of sepsis is severe viral infection and stimulates the body's immune response, causing the release of a large number of immune factors [5, 6]. Therefore, it will cause different systems and organs throughout the body to varying degrees, and the impact of immune disorders will eventually harm the human body. Sepsis is still one of the diseases with a high mortality rate in the intensive care unit, and it is a severe challenge facing the medical department. According to relevant adult studies, the incidence of sepsis in adults is increasing year by year, and the mortality rate remains at a high level of 30% to 50% [7, 8]. Based on child-related survey data, the prevalence of sepsis in the pediatric intensive care unit is about 17%, and the mortality rate of severe sepsis is about 10% to 48% [9–10]. If patients with sepsis are not properly treated, they will gradually develop into multiple organ failure syndrome, which seriously threatens the children's lifelong health. At present, there are many studies on the causes and harmful factors of sepsis at home and abroad, but the results are relatively single. Sepsis can be caused by infection in any part. Clinically, it is common in pneumonia, peritonitis, cholangitis, urinary system infection, cellulitis, meningitis, abscess, and so on. Pathogenic microorganisms include bacteria, fungi, viruses, and parasites, but not all patients with sepsis have positive blood culture results of pathogenic microorganisms causing infection.

This article combines the clinical data of children with PICU sepsis admitted to a hospital from January 2016 to January 2019, divides the children into death groups and survival groups, and analyzes their clinical characteristics and death risk factors. All the data was analyzed by SPSS21.0 statistical analysis software. The fundamental pathogenesis of sepsis is not yet clear, which involves complex systemic inflammatory network effects, gene polymorphisms, immune dysfunction, abnormal coagulation function, tissue damage, and abnormal host response to different infectious pathogenic microorganisms and toxins. It is closely related to the pathophysiological changes of multiple systems and organs. The pathogenesis of sepsis still needs to be further clarified.

## 2. Clinical Characteristics and Death Risk Factors of Severe Sepsis in Children

### 2.1. The Pathogenesis of Sepsis

#### 2.1.1. Blood Coagulation Dysfunction

DIC is the most serious plasma coagulation disease, and it is one of the main mechanisms for the development of MODS sepsis. The DIC branch of the ISTH Scientific Standards Committee focuses on the damage and inflammation of the capillary endothelium and defines the sepsis induced by DIC. In sepsis, due to the large amount of excretion of various proinflammatory and anti-inflammatory drugs, it will affect the plasma coagulation system. At the same time, because the normal antifreeze cells and fibrinolytic system are inhibited to varying degrees, the blood tends to become hypercoagulable, which also causes cerebral embolism and circulatory dysfunction in microvessels and small blood vessels, and more severe sepsis, dan toxic shock, etc., eventually evolved into MODS [11, 12].

#### 2.1.2. Bacterial Infection

Both bacterial and fungal infections can form sepsis. Among them, bacterial infections are more commonly caused by coagulation-negative Staphylococcus aureus. In recent years, due to the large-scale application of antibiotics, the pathogenic bacteria that cause sepsis are not limited to pathogenic particles, bacilli, and fungi. The gram-negative bacteria that cause spoilage are mainly in the Enterobacteriaceae, among which are Escherichia coli infection, Klebsiella bacteria, and Pseudomonas aeruginosa, among which Escherichia coli infection is more common.

#### 2.1.3. Apoptosis

Multiple organ failure caused by sepsis is mainly due to the conversion of cells to an anti-inflammatory phenotype. Apoptosis, abbreviated as programmed cell apoptosis, is an active cell apoptosis process regulated by genes, including the development of multicellular individuals and the maintenance of internal environment stability. The apoptosis of mononuclear macrophages and T and B lymphocytes are all involved in the pathological process of sepsis and septic shock.

#### 2.1.4. Innate Immunity and Cytokines

Innate immunity is also called nonspecific or innate immunity. The body exerts its initial anti-infection function through immune response, which is a “hard sword.” Overactivated immune cells, the cytokines they produce, and the active ingredients of supplements can damage normal tissue cells. The damage of various cytokines in endothelial cells and solid organs after purulent bacterial infection is the main cause of septic shock. In the early stages of sepsis, blood cytokines are TNF-*α*, IL-6, and IL-8. Significant increase in many inflammatory response factors can lead to cardiovascular dysfunction, thereby promoting the deterioration of sepsis and multiple organ failure. Therefore, suppression of inflammatory response is the focus of sepsis treatment.

Gene polymorphism: the clinical manifestations and prognosis of different individuals commonly infected with the same pathogen are quite different, suggesting that genetic factors such as gene polymorphism are also important factors affecting human susceptibility and tolerance to stress, diversity of clinical manifestations, and differences in drug treatment response.

### 2.2. Treatment of Septic Shock

#### 2.2.1. Replenish Blood Volume

It mainly provides crystals, colloidal solutions, and blood products for reducing swelling. After fluid replacement, the response to treatment depends on increased blood pressure, decreased heart rate, improved response, peripheral vasoconstriction, and restoration of urine supply. If the patient is satisfied with the hydration response and does not have pulmonary edema, there is no need to use vasoactive drugs or invasive monitoring devices.

#### 2.2.2. Vasoactive Drugs

Patients with severe sepsis and shock may have low excretion and high resistance, high excretion and low resistance, or even low excretion and low resistance. In various stages of severe sepsis or in different treatment periods, hemodynamic conditions may change to different conditions. Therefore, exercise enhancers and inotropic drugs should be selected according to the child's clinical condition. The correct use of vasoactive agents should be confirmed by laboratory testing.

#### 2.2.3. Antibiotic Treatment

Early and prompt antibiotic treatment of severe sepsis and septic shock requires intravenous antibiotics within 1 hour of diagnosis. Intravenous antibiotics can quickly reach a certain level in the blood. This is an effective way to prevent bacterial shock in the body. Early use of antibiotics and fluid recovery are also very important.

#### 2.2.4. Obtain Biological Evidence

As far as possible, biological samples shall be taken before the use of antibiotics for bacterial/fungal culture. The samples include blood, sputum, urine, wound secretion, and other samples. The culture results are conducive to the targeted use of antibiotics, but not all biological specimen cultures of sepsis will have positive results.

## 3. Experiment

### 3.1. Objects

This article selects the clinical data of children with PICU sepsis admitted to a hospital from January 2016 to January 2019. A total of 65 cases were collected, of which 8 cases had basic cases, 41 males, 24 females, and 29 were transferred from the hospital. 36 cases were transferred from outside hospitals or directly into PICU. Among them, 15 cases died in the hospital, 22 cases were improved and discharged, and 28 cases were discharged from the hospital by signing.

### 3.2. Diagnostic Criteria

The diagnostic criteria for childhood sepsis and severe sepsis refer to the criteria jointly formulated by the American Thoracic Society/Emergency Medical Association in 2005.

### 3.3. Clinical Data

#### 3.3.1. Infection

The 65 children with severe sepsis who participated in the study denied any history of allergies, trauma, stress, immunosuppressants, and chemotherapy drugs. The clinical symptoms of SIRS are mainly manifested as changes in respiratory frequency and heart rate, accompanied by fever or abnormal white blood cell counts in blood tests, etc., and relevant imaging examinations and causal testing of the infected site are required to determine the treatment of infection. Systemic inflammatory response syndrome refers to systemic inflammatory response. Endotoxin is the trigger of systemic inflammatory response, and there is no obvious drug cure. On the one hand, inflammatory cells can activate granulocytes to damage endothelial cells, platelet adhesion, release oxygen free radicals, and lipid metabolites; on the other hand, they can further promote the activation of inflammatory cells. The two are cause and effect, and form a “waterfall effect” in the body, resulting in the continuous increase of the number of inflammatory mediators and the continuous expansion of inflammatory response. When the body's compensatory capacity is exceeded, the body has excessive inflammatory response, causing extensive tissue and cell damage, resulting in systemic inflammatory cell response syndrome.

#### 3.3.2. Severe Case Score PCIS in Children

Ten items of vital signs (respiration, heart rate, blood pressure), liver function, blood gas analysis, water and electrolyte balance, etc. were evaluated when the child entered PICU, and the score was defined as 80-71 as critical; score ≤ 70 was extremely severe critically.

### 3.4. Statistical Analysis

SPSS is the earliest statistical software in the world that uses graphical menu driven interface. Its most prominent feature is that the operation interface is very friendly, and the output results are beautiful. It shows almost all functions in a unified and standardized interface and uses the windows window to show the functions of various data management and analysis methods, and the dialog box shows various function options. It integrates the functions of data entry, sorting, and analysis. Users can select modules according to actual needs and computer functions, so as to reduce the requirements for the capacity of system hard disk, which is conducive to the popularization and application of the software. The basic functions of SPSS include data management, statistical analysis, chart analysis, and output management. Use SPSS21.0 statistical analysis software for statistical analysis. The description of the measurement data is usually represented by $\left(\bar{X}\pm s\right)$. If the two measurement data meet the normal distribution and the variances are equal, the independent sample *t*-test can be used. Count data is generally described by the composition of percentage (%), while the second count data is generally tested by *χ*^2^. *P* < 0.05 is considered statistically significant. The *t*-test calculation formula is

(1) $$\begin{array}{c} t=\frac{\bar{X}-\mu }{\sigma_{X}/\sqrt{n-1}}. \end{array}$$

If the sample is a large sample, it can also be written as

(2) $$\begin{array}{c} t=\frac{\bar{X}-\mu }{\sigma_{X}/\sqrt{n}}. \end{array}$$

Here, *t* is the deviation statistic between the sample mean and the population mean; $\bar{X}$ is the sample mean.

The graphic features of the normal distribution curve include concentration: the peak of the normal curve is located in the positive center, that is, the position of the mean; symmetry: the normal curve is centered on the mean, symmetrical left and right, and the two ends of the curve will never intersect the horizontal axis; and uniform variability: the normal curve starts from the place where the mean is located and gradually decreases evenly to the left and right sides, respectively.

## 4. Discussion

### 4.1. Clinical Characteristics

#### 4.1.1. General Situation

From 2016 to 2019, a PICU in a hospital admitted 65 children with severe sepsis. The incidence rate was 3.8%, and the average age of onset was 314.6 days. Children younger than 1 year accounted for 53.8% (35/65): male children 63.1% (41/65) and female children 36.9% (24/65). Eight of the 65 children had basic cases, accounting for 12.3%. There were 34 children with shock, accounting for 52.3%, and 43 children with MODS, accounting for 66.2%. Of the 65 children, 15 died in the hospital, with a fatality rate of 23.1%. The details are shown in Table 1 and Figure 1.

#### 4.1.2. Etiology

Among 65 children with severe sepsis, 29.2% (19/65) had the respiratory tract as the primary infection, 32.3% (21/65) had the digestive system, and 15.4% (10/65) had intracranial infection. At the same time, the respiratory system and the digestive system are 7.7% (5/65) of the primary lesions.

It can be seen from Table 2 and Figure 2 that among the 65 cases of severe sepsis, 19 cases have the respiratory tract as the primary infection, accounting for 29.2%, and 21 cases have the digestive system, accounting for 32.3%. There were 10 cases of internal infection, accounting for 15.4%, 5 cases with respiratory system and digestive system as primary foci, accounting for 7.7%, and 6 cases of skin and soft tissue infection, accounting for 9.2%.

#### 4.1.3. Supportive Treatment

Among all included statistics, 47 cases of severe sepsis used mechanical ventilation, accounting for 72.3%. The average ventilation time was 97 hours, and 12 cases died, accounting for 25.5%. Among them, 31 cases of mechanical ventilation time were more than 24 hours, and deaths occurred, 5 cases, accounting for 16.1%. Twenty patients who used continuous blood purification accounted for 30.8%, and 3 patients (15%) died. There were 43 cases (66.2%) using vasoactive drugs, and 11 cases (25.6%) died. 22 cases of children used gamma globulin, accounting for 33.8%. There are 54 cases (83.1%) of children who received blood component transfusion. Details are shown in Table 3 and Figure 3. Mechanical ventilation-assisted ventilation: in case of acute lung injury/acute respiratory distress syndrome in patients with severe sepsis, mechanical ventilation treatment should be carried out in time to alleviate tissue hypoxia, and it is suggested to choose the protective lung ventilation strategy of low plateau pressure, low tidal volume ventilation, and permissive hypercapnia.

### 4.2. Risk Factors for Death from Severe Sepsis in Children

#### 4.2.1. Single Factor Analysis

For factors such as gender, age, WBC absolute value count, neutrophil absolute value count, http://HB.PLT.CRALT.TP value, ALB, CRP, arteriole blood pH, PO2, PCO2, and BE, single-cause conditions have been developed logistic regression analysis, and according to the level of *a* = 0.05, selected eight kinds of significant statistically significant influencing factors. The detailed data of the eight variables directly related to the mortality of severe sepsis are shown in Table 4 and Figure 4.

#### 4.2.2. Multifactor Analysis

It can be seen from Table 5 that there are eight main influencing factors that have major statistical significance in the results of single factor analysis. Therefore, the following describes the unconditional logistic regression analysis of their influence. Among them, serum lactate value, PCIS value and MODS value, and the removal factors of the three indicators of the number of organs involved have a greater impact on the interaction, but they are also directly related to the high mortality rate of severe pediatric sepsis. It should be noted that the new diagnostic criteria do not emphasize that sepsis can be diagnosed only by adding the above 5 or more manifestations on the basis of infection, but more emphasize to make a clinical diagnosis of sepsis more in line with the clinical reality with abnormal indicators combined with the specific condition changes of clinical specialties.

## 5. Conclusions

Sepsis is a common disease in pediatrics, with rapid development and rapid progress, becoming a serious disease. When it appears, it consumes more human and material resources and may not produce satisfactory results. Therefore, this article summarizes the related factors of death from sepsis and the contribution of corresponding treatments in reducing the mortality rate. It is hoped that the disease can be better diagnosed, and appropriate treatments can be used to help prevent the disease from further developing into severe or septic shock and to prevent the disease from further developing into severe or septic shock. Patients who have been combined with MODS or septic shock should receive early treatment and reasonable diagnosis in order to improve the prognosis and reduce the mortality rate.

## Figures and Tables

**Figure 1:** General situation.

**Figure 2:** Primary infection.

**Figure 3:** Related therapeutic effects.

**Figure 4:** Univariate variables associated with death from severe sepsis.

**Table 1:** General situation.

	PICU included cases	Death
Total	65	15
12.3	41	9
Number of female cases	24	6
Number of basic cases	8	5
Combined shock cases	34	8
Number of combined MODS cases	43	10

**Table 2:** Primary infection.

Primary infection	Number of cases	Percentage
Respiratory tract infection	19	29.2%
Digestive tract infection	21	32.3%
Intracranial infection	10	15.4%
Simultaneous respiratory and digestive tract infections	5	7.7%
Skin and soft tissue infections	6	9.2%
Other	4	6.2%
Total	65	100%

**Table 3:** Related therapeutic effects.

	Survive	Death
Mechanical ventilation	35	12
Mechanical ventilation time is greater than 24 hours	26	5
Continuous blood purification	17	3
Use of vasoactive drugs	32	11

**Table 4:** Univariate variables associated with death from severe sepsis.

Influencing factors		Nondeath group (*n* = 50)	*B*	SE	Wald *χ*^2^	*P*	OR
Low blood pressure		1	4.126	1.102	14.005	0.000	62.011
Mechanical ventilation		35	3.566	1.058	11.334	0.001	35.408
Serum lactate value		4.07 ± 0.74	0.165	0.052	9.794	0.002	1.180
Hemoglobin		102.84 ± 15.33	0.026	0.011	4.893	0.026	0.973
Total protein		58.67 ± 7.46	0.059	0.027	4.575	0.031	0.941
Albumin		37.92 ± 5.47	0.096	0.441	5.232	0.021	0.907
PCIS		84.07 ± 6.03	0.179	0.046	14.668	0.000	0.834
Number of organs involved in MODS	<3	48	2.724	0.575	19.254	0.000	15.250
	≥3	2					

**Table 5:** Multivariate unconditional logistic regression analysis.

Influencing factors		Death group (*n* = 15)	Nondeath group (*n* = 50)	*B*	SE	Wald *χ*^2^	*P*	OR
Low blood pressure		7	1	15.068	89.977	0.027	0.866	3401062
Mechanical ventilation		12	35	6.166	3.401	3.285	0.069	475.64
Serum lactate value		8.21 ± 1.64	4.07 ± 0.74	-1.468	0.725	4.095	0.042	0.221
Hemoglobin		89.25 ± 30.25	102.84 ± 15.33	-0.378	0.168	4.493	0.061	0.729
Total protein		52.41 ± 11.86	58.67 ± 7.46	-0.297	0.378	0.618	0.430	0.741
Albumin		34.05 ± 7.82	37.92 ± 5.47	0.34	0.575	0.359	0.452	1.418
PCIS		73.19 ± 7.14	84.07 ± 6.03	-0.668	0.371	3.059	0.038	2.642
Number of organs involved in MODS	<3	3	48	11.757	4.624	4.624	0.031	126882.4
	≥3	12	2					

## Data Availability

The data underlying the results presented in the study are available within the manuscript.
